The article "Long non-coding RNA linc-ITGB1 promotes cell proliferation, migration, and invasion in human hepatoma carcinoma by up-regulating ROCK1" was retracted in 2023. Reasons: errors in the materials; concerns about the data.

# Long non-coding RNA linc-ITGB1 promotes cell proliferation, migration, and invasion in human hepatoma carcinoma by up-regulating ROCK1

**DOI:** 10.1042/BSR20181289

**Published:** 2018-10-31

**Authors:** Lei Huang, Xinyu Li, Weijie Gao

**Affiliations:** Department of Hepatobiliary Surgery, Peking University People’s Hospital, Beijing 100044, P.R. China

**Keywords:** hepatoma carcinoma, invasion, Linc-ITGB1, migration, proliferation, ROCK1

## Abstract

**Background:** Linc-ITGB1 is a newly identified long non-coding RNA (lncRNA) involved in the regulation of cell migration and invasion of gallbladder cancer cell lines, while its involvement in human hepatoma carcinoma (HCC) is unknown. **Methods:** In the present study, HCC patient tumor tissues, adjacent healthy tissues and whole blood were collected from both HCC patients and healthy controls. Expression of LINC-ITGB1 was examined by qRT-PCR. Diagnostic value of serum LINC-ITGB1 for HCC was evaluated by receiver operating characteristic (ROC) curve analysis. Correlation between the serum LINC-ITGB1 and basic clinical information of patients was analyzed by chi-square test. LINC-ITGB1 overexpression HCC cell lines were established and the effects on cell proliferation, migration, and invasion were explored by CCK-8 assay and Transwell assay. Effects of LINC-ITGB1 overexpression on Rho-associated, coiled-coil-containing protein kinase 1 (ROCK1) expression were investigated by Western blot. **Results:** We found that LINC-ITGB1 was up-regulated in tumor tissues than in adjacent healthy tissues. Serum levels of LINC-ITGB1 were higher in HCC patients than in healthy controls. Serum levels of LINC-ITGB1 were significantly correlated with tumor size and distant tumor metastasis. LINC-ITGB1 overexpression promoted the proliferation, migration, and invasion of HCC cells and the expression of ROCK1. ROCK1 inhibitor reduced the effects of LINC-ITGB1 overexpression on cell proliferation, migration, and invasion. **Conclusion:** We conclude that lncRNA LINC-ITGB1 can promote the proliferation, migration, and invasion of HCC cells by up-regulating ROCK1.

## Background

It is generally believed that liver cancer is the ninth most common malignancy in females and fifth most common malignancy in males; due to the high mortality rate, liver cancer ranks second amongst all causes of cancer-related deaths [1]. In recent years, incidence of liver cancer shows an increasing trend, especially in developing countries such as China, disease burden of liver cancer is increasing every year [2]. As the most common type of liver cancer, human hepatocellular carcinoma (HCC) is mainly caused by chronic liver inflammation and chronic viral hepatitis infection [3]. At present, treatment of HCC is still challenged by the existing distant tumor metastasis by the time of diagnosis [4]. Therefore, early diagnosis and treatment is still critical for the survival of HCC patients.

The article "Long non-coding RNA linc-ITGB1 promotes cell proliferation, migration, and invasion in human hepatoma carcinoma by up-regulating ROCK1" was retracted in 2023. Reasons: errors in the materials; concerns about the data.

Hepatitis B virus (HBV) infection and the development of HCC are accompanied with changes in a large set of genes including non-coding RNAs [5]. Linc-ITGB1 is a newly identified long non-coding RNA (lncRNA) involved in the regulation of cell migration and invasion of gallbladder cancer [6] and breast cancer [7]. However, its involvement in other malignancies is unknown. Rho-associated, coiled-coil-containing protein kinase 1 (ROCK1) participates in the regulation of cell motility, metastasis, and angiogenesis during the development of malignancies [8]. It is reported that ROCK1 may interact with lncRNAs to participate in tumor development [9]. Therefore, it would be of great interest to explore the functionality of linc-ITGB1 and ROCK1 as well as the possible interactions between them. In our study, we found that Linc-ITGB1 can promote the proliferation, migration, and invasion of HCC cells by up-regulating ROCK1, which might provide new insights into the treatment of HCC.

## Materials and methods

### Subjects

Our study included 80 patients with HCC. Those patients were diagnosed as HCC through pathological examinations and treated from January 2016 to January 2018 in Peking University People’s Hospital for the first time. Patients with other liver diseases, other types of malignancies, and other severe diseases were excluded. Patients who were treated in other hospitals before admission were not included. Those patients included 47 males and 33 females, and age ranged from 33 to 69 years, with an average of 50.2 ± 7.4 years. Distant tumor metastasis was found in 33 patients. Our study also included 44 healthy volunteers to serve as a control group. All healthy volunteers were confirmed with normal physiological conditions in our hospital. Control group included 24 males and 20 females, and age ranged from 29 to 66 years, with an average of 48.9 ± 10.1 years. There were no significant differences in age and gender between two groups. The study was approved by the Ethics Committee of Peking University People’s Hospital. All patients signed informed consent.

### Specimen collection

Amongst 80 HCC patients, 56 patients received surgical resection of tumors and other patients were treated with other treatment due to severe conditions that were not suitable for surgery. Tumor tissues and adjacent healthy tissues were obtained from those 56 HCC patients during surgical operations. Besides that, blood (approximately 10 ml) was collected from the elbow vein of all 80 patients with HCC and 44 healthy controls. Blood was kept at 37°C for 2 h, followed by centrifugation at 1875 rpm for 20 min to obtain serum. All tissues were stored in liquid nitrogen before use.

The article "Long non-coding RNA linc-ITGB1 promotes cell proliferation, migration, and invasion in human hepatoma carcinoma by up-regulating ROCK1" was retracted in 2023. Reasons: errors in the materials; concerns about the data.

### Cell lines and cell culture

Human HCC cell lines C3A (CRL10742™) and HEP G2 (CRL11997™), as well as a normal liver tissue cell line THLE-3 (ATCC® CRL-11233™) were provided by American Type Culture Collection (ATCC, U.S.A.). Cells were cultured in DMEM containing 10% FBS (Invitrogen, Carlsbad, CA), 100 mg/ml penicillin G (Invitrogen, Carlsbad, CA), and 100 U/ml streptomycin (Invitrogen, Carlsbad, CA) in an incubator (37°C, 5% CO_2_). FBS was not added in ROCK1 inhibitor treatment experiments.

### Real-time quantitative PCR

Total RNA extraction from *in vitro* culture cells, serum, tumor tissues, and adjacent healthy tissues was performed using TRIzol reagent (Invitrogen, U.S.A.). Tumor tissues and adjacent healthy tissues were ground in liquid nitrogen before the addition of Trizol reagent. cDNA was synthesized using AMV reverse transcriptase (GIBCO, U.S.A.) through reverse transcription. PCR were performed using following primers: 5′-CCTCTCAGCCTCCAGCGTTG-3′ (forward) and 5′-TGCTCTTGCTCACTCACACTCC-3′ (reverse) for linc-ITGB1; 5′-CAGGAGGCATTGCTGATGAT-3′ (forward) and 5′-GAAGGCTGGGGCTCATTT-3′ (reverse) for GAPDH. Relative expression levels of linc-ITGB1 were normalized to endogenous control GAPDH using 2**^−^**^ΔΔ*C*^_T_ methods. All PCR products were subjected to 2% agarose gel electrophoresis and only one band was observed. This experiment was performed in triplicate manner and data were expressed as mean ± S.D.

### Cell transfection

Full-length linc-ITGB1 cDNA was cloned into pcDNA3.1 vector to make linc-ITGB1 expression vector. LINC-ITGB1 shRNA (5′-GCAGCTGTTTCCAGAATATTGCTCGAGCAATATTCTGGAAACAGCTGC-3′) and negative control shRNA (5′-GCGGAGGGTTTGAAAGAATATCTCGAGATATTCTTTCAAACCCTCCGCTTTTTT-3′) were synthesized by GenePharma (Shanghai, China). Lipofectamine 2000 (11668-019, Invitrogen, Carlsbad, U.S.A.) was used for the transfection of vectors and shRNAs at a dose of 10 and 50 nM, respectively. Cells without transfection were used as negative control. Expression of Linc-ITGB1 was detected before each experiment by qRT-PCR. Subsequent experiment was only performed in case of overexpression rate above 200% and knockdown rate below 50% compared with control cells was achieved.

### Cell proliferation assay

CCK-8 assay was used to detect cell proliferation; 4 × 10^3^ cells in 100 μl culture medium were added to each well of 96-well plate. Cells were cultured at 37°C (5% CO_2_), and 10 μl of CCK-8 solution was added into each well 12, 24, 48, and 96 h later. Cells were cultured for another 4 h, and OD values at 450 nm were measured using Fisherbrand™ accuSkan™ GO UV/Vis Microplate Spectrophotometer (Fisher Scientific). This experiment was performed in triplicate manner and data were expressed as mean ± S.D.

The article "Long non-coding RNA linc-ITGB1 promotes cell proliferation, migration, and invasion in human hepatoma carcinoma by up-regulating ROCK1" was retracted in 2023. Reasons: errors in the materials; concerns about the data.

### Transwell migration and invasion assay

Cell suspension was prepared with a final density of 5 × 10^4^ cells/ml. For Transwell migration assay, 4 × 10^4^ cells in 0.1 ml serum-free culture medium were transferred to the upper chamber, and RPMI-1640 medium (Thermo Fisher Scientific, U.S.A.) containing 20% FCS (Sigma–Aldrich, U.S.A.) was added into the lower chamber. Cells were cultured for 24 h and membranes were collected, cleaned, and stained with 0.5% Crystal Violet (Sigma–Aldrich, U.S.A.) at room temperature for 30 min. For invasion assay, upper chamber was coated with Matrigel (356234, Millipore, U.S.A.) before adding cells. Cell migration and invasion was normalized to cell proliferation data at 24 h to avoid the effects from cell proliferation. This experiment was performed in triplicate manner and data were expressed as mean ± S.D.

### Western blot

Total protein extraction from *in vitro* cultured cells was performed using cell lysis buffer (P0013K, Beyotime), and protein concentration was measured using BCA assay. SDS/PAGE (10% gel) was performed to separate proteins. After gel transfer, PVDF membranes were blocked with 5% skimmed milk at room temperature for 1 h, followed by incubation with primary antibodies including rabbit anti-ROCK1 (1:1500, ab45171, Abcam) and rabbit anti-β-actin (1:1500, ab8227, Abcam) overnight at 4°C. Membranes were washed with TBST (0.3% Tween20), followed by incubation with anti-rabbit IgG-HRP secondary antibody (1:1000, MBS435036, MyBioSource) at room temperature for 2 h. After washing with TBST (0.3% Tween20), ECL (Sigma–Aldrich, U.S.A.) method was used to develop signals, and relative expression level of ROCK1 was normalized to endogenous control β-actin using ImageJ V1.6. This experiment was performed in triplicate manner and data were expressed as mean ± S.D.

### Statistical analysis

SPSS19.0 (SPSS Inc., U.S.A.) was used in the present study to analyze all data. Comparisons between two groups or amongst multiple groups were performed by unpaired *t*test and one-way ANOVA followed by LSD test, respectively. *P*<0.05 was considered to be statistically significant.

### Availability of data and materials

Please contact authors for data request.

## Results

### Expression of linc-ITGB1 in HCC tissues and adjacent healthy tissues in 56 HCC patients

Expression of linc-ITGB1 in HCC tissues and adjacent healthy tissues of 56 patients with HCC was examined by qRT-PCR. As shown in Figure 1, expression level of linc-ITGB1 was significantly higher in HCC tissues than in adjacent healthy tissues in 52 out of 56 patients (*P*<0.05). In contrast, only two patients showed lower expression levels of linc-ITGB1 in HCC patients than in healthy controls. Our data may indicate that up-regulation of linc-ITGB1 is very likely involved in the pathogenesis of HCC.

The article "Long non-coding RNA linc-ITGB1 promotes cell proliferation, migration, and invasion in human hepatoma carcinoma by up-regulating ROCK1" was retracted in 2023. Reasons: errors in the materials; concerns about the data.

**Figure 1:** Expression of linc-ITGB1 in HCC tissues and adjacent healthy tissues in 56 HCC patients Expression level of linc-ITGB1 was significantly higher in HCC tissues than in adjacent healthy tissues in 52 out of 56 patients. *Compared with adjacent healthy tissue, *P*<0.05; compared with HCC tissues, *P*<0.05.

### Serum levels of linc-ITGB1 in HCC patients and healthy controls and the diagnostic values

qRT-PCR results showed that serum levels of linc-ITGB1 were significantly higher in HCC patients (*n*=80) than in healthy controls (*n*=44) (Figure 2A). Receiver operating characteristic (ROC) curve analysis was performed to evaluate the diagnostic value of linc-ITGB1 for HCC. As shown in Figure 2B, the area under the curve (AUC) is 0.8520 with 95% confidence interval of 0.7840–0.9200 (*P*<0.0001). Our data may suggest that up-regulation of linc-ITGB1 can be a potential diagnostic marker for HCC.

**Figure 2:** Serum levels of linc-ITGB1 in HCC patients and healthy controls and diagnostic values (**A**) Level of linc-ITGB1 in serum of healthy controls and patients with HCC. (**B**) ROC curve of the use of linc-ITGB1 in the diagnosis of HCC. Serum levels of linc-ITGB1 were significantly higher in HCC patients than in healthy controls and the high serum levels of linc-ITGB1 distinguished HCC patients from healthy controls. *, *P*<0.05

### Correlations between serum levels of linc-ITGB1 and clinicopathological data of HCC patients

Eighty patients with HCC were divided into high and low expression groups according to the median serum levels of linc-ITGB1 (*n*=40). Correlations between serum levels of linc-ITGB1 and clinicopathological data of HCC patients were analyzed by Chi-square test. In the present study, distant metastasis was observed in 33 patients, including 22 cases of lung metastasis and 11 cases of bone metastasis. As shown in Table 1, serum levels of linc-ITGB1 were not significantly correlated with patients’ gender, age, smoking, and drinking habits, but were significant correlated with tumor size, distant metastasis, and AJCC stage.

**Table 1:** Correlations between serum levels of linc-ITGB1 and clinicopathological data of HCC patients

Items	Groups	Cases	High expression	Low expression	χ^2^	*P*-value
Gender	Male	47	22	25	0.46	0.5
	Female	33	18	15		
Age (years)	>50	39	17	22	1.25	0.26
	<50	41	23	18		
Primary tumor diameter (cm)	>5	45	31	14	14.68	0.0001
	≤5	35	9	26		
Tumor distant metastasis	Yes	33	22	11	6.24	0.12
	No	47	18	29		
AJCC stage	I–II	22	8	14	12.29	0.0005
	III–IV	58	32	26		
Smoking	Yes	48	22	26	0.83	0.36
	No	32	18	14		
Drinking	Yes	46	20	26	1.84	0.17
	No	34	20	14		

The article "Long non-coding RNA linc-ITGB1 promotes cell proliferation, migration, and invasion in human hepatoma carcinoma by up-regulating ROCK1" was retracted in 2023. Reasons: errors in the materials; concerns about the data.

### Effects of linc-ITGB1 overexpression on ROCK1 expression

ROCK1 plays an important role in the growth and metastasis of tumors, and inhibition of ROCK1 is considered to be a promising target for the treatment of various types of tumors including HCC [10]. To test whether linc-ITGB1 regulates ROCK1 expression, linc-ITGB1 expression vector or shRNA was transfected into cells of HCC cell lines C3A and HEP G2, as well as a normal liver tissue cell line THLE-3. Overexpression and knockdown of linc-ITGB1 were confirmed by qRT-PCR. As shown in Figure 3A, linc-ITGB1 overexpression and knockdown were reached after transfection. Overexpression of linc-ITGB1 led to significantly up-regulated expression of ROCK1 in cells of HCC cell lines C3A and HEP G2 (Figure 3B, *P*<0.05), but not in normal liver tissue cell line THLE-3. In contrast, linc-ITGB1 knockdown significantly down-regulated the expression of ROCK1 in HCC cell lines C3A and HEP G2 (*P*<0.05), but not in normal liver tissue cell line THLE-3 (Figure 3C).

**Figure 3:** Effects of linc-ITGB1 overexpression and knockdown on ROCK1 expression Linc-ITGB1 overexpression and knockdown were reached after transfection (**A**). Linc-ITGB1 overexpression significantly up-regulated (**B**), while linc-ITGB1 knockdown (**C**) significantly down-regulated the expression of ROCK1 in cells of HCC cell lines C3A and HEP G2 but not in normal liver tissue cell line THLE-3. *, *P*<0.05.

### Effects of linc-ITGB1 overexpression on HCC cell proliferation, migration, and invasion

Data listed in Table 1 showed that up-regulation of linc-ITGB1 is very likely involved in the growth and metastasis of HCC. Therefore, we further investigated the effects of linc-ITGB1 overexpression on proliferation, migration, and invasion of HCC cells. Expression level of Linc-ITGB1 was significantly higher in C3A and HepG2 than in THLE-3 (data not shown). As shown in Figure 4, linc-ITGB1 overexpression significantly promoted the proliferation (Figure 4A), migration (Figure 4B), and invasion (Figure 4C) in cells of HCC cell lines C3A and HEP G2 (*P*<0.05). However, treatment with Stemolecule™ ROCK I Inhibitor (10 nM, CAS# 203911-26-6, Stemgent Inc.) for 12 h significantly reduced the enhancing effects of linc-ITGB1 overexpression on proliferation (Figure 4A), migration (Figure 4B), and invasion (Figure 4C) of HCC cells (*P*<0.05). In contrast, linc-ITGB1 knockdown significantly inhibited the proliferation (Figure 5A), migration (Figure 5B), and invasion (Figure 5C) of HCC cell lines C3A and HEP G2 (*P*<0.05). In addition, linc-ITGB1 overexpression, linc-ITGB1 knockdown, and temolecule™ ROCK I Inhibitor showed no significant effects on cells of normal liver tissue cell line THLE-3 (*P*>0.05).

The article "Long non-coding RNA linc-ITGB1 promotes cell proliferation, migration, and invasion in human hepatoma carcinoma by up-regulating ROCK1" was retracted in 2023. Reasons: errors in the materials; concerns about the data.

**Figure 4:** Effects of linc-ITGB1 overexpression on HCC cell proliferation, migration, and invasion This figure shows proliferation (**A**), migration (**B**), and invasion (**C**) of two HCC cell lines C3A and HEP G2 and a normal liver tissue cell line THLE-3 under linc-ITGB1 overexpression and ROCK1 inhibitor treatment. Linc-ITGB1 overexpression significantly promoted the proliferation, migration, and invasion of HCC cell lines C3A and HEP G2 but not normal cell line THLE-3. Treatment with Stemolecule™ ROCK I Inhibitor significantly reduced the enhancing effects of linc-ITGB1 overexpression on cancer cell proliferation, migration, and invasion of HCC cells. *, *P*<0.05; IH, ROCK1 inhibitor.

**Figure 5:** Effects of linc-ITGB1 knockdown on HCC cell proliferation, migration, and invasion This figure shows proliferation (**A**), migration (**B**), and invasion (**C**) of two HCC cell lines C3A and HEP G2 and a normal liver tissue cell line THLE-3 under linc-ITGB1 knockdown. Linc-ITGB1 knockdown significantly inhibited cancer cell proliferation, migration, and invasion, but showed no significant effects on cells of normal liver tissue cell line THLE-3. *, *P*<0.05.

## Discussion

In the present study, we reported that linc-ITGB1 as a newly identified lncRNA with unknown functionality in most types of malignancies is involved in the regulation of proliferation, migration, and invasion of HCC cells. We also provided evidence that the function of linc-ITGB1 in HCC is likely, at least partially, achieved through the up-regulation of ROCK1.

Changes in expression pattern of a large set of lncRNAs have been observed during the onset, development, and progression of HCC [11]. As an oncogenic lncRNA, UCA1 is highly expressed in HCC tissues than in adjacent healthy liver tissues, and the up-regulation of UCA1 has been proved to be correlated with the progression of HCC and poor prognosis after treatment [12]. In contrast, down-regulation of lncRNA GAS5 is observed during the development of HCC, indicating its role as a tumor suppressor lncRNA in HCC [13]. Linc-ITGB1 overexpression has been observed in gallbladder cancer [6] and breast cancer [7]. In this study, up-regulated expression of linc-ITGB1 was observed in 52 out of 56 HCC patients, accounting for 92.9% of all cases, indicating that linc-ITGB1 may also play a role as tumor suppressor gene in HCC.

The article "Long non-coding RNA linc-ITGB1 promotes cell proliferation, migration, and invasion in human hepatoma carcinoma by up-regulating ROCK1" was retracted in 2023. Reasons: errors in the materials; concerns about the data.

Treatment of HCC is still challenged by the existence of distant tumor metastasis by the time of diagnosis and early diagnosis is still critical. Changes in levels of certain substances in blood were usually observed during the development of human diseases, and monitoring the blood levels of those substances may provide important guidance for the treatment of those diseases [14]. In our study, significantly higher serum levels of linc-ITGB1 were observed in HCC patients compared with healthy controls. Furthermore, ROC curve analysis also showed that serum linc-ITGB1 can be used to effectively distinguish HCC patients from healthy controls, indicating the potential application of serum linc-ITGB1 as a diagnostic marker for HCC. It has been well established that ageing, smoking habit, alcohol abuse, and other factors affect the expression pattern of certain lncRNAs [15–17]. In this study, serum levels of linc-ITGB1 showed no significant correlations with age, gender as well as patients’ smoking and drinking habits. Therefore, the use of linc-ITGB1 in the diagnosis will not be affected by those individuals’ backgrounds, indicating the high reliability.

Our study also showed that serum levels of linc-ITGB1 were significantly correlated with tumor size and distant tumor metastasis. Our experiments at cellular level also showed that linc-ITGB1 overexpression promoted proliferation, migration as well as invasion of HCC cells. ROCK1 has diverse functions in the human body. Activation of ROCK1 is involved in the development of human malignancies [18], and inhibition of ROCK1 now is considered to be a potential therapeutic target for the treatment of different types of human malignancies [19,20]. In a recent study, ROCK was shown to interact with JAK1 signaling to participate in the regulation of tumor metastasis through by controlling actomyosin contractility [21]. In our study, linc-ITGB1 overexpression significantly up-regulated the expression of ROCK1 in cells of two HCC cell lines, and ROCK1 inhibitor treatment reduced the enhancing effects of ROCK1 overexpression on HCC cell proliferation, migration, and invasion, suggesting that linc-ITGB1 may activate ROCK1 to promote HCC growth and metastasis. It is also noteworthy that linc-ITGB1 and ROCK1 inhibitor treatment showed no significant effects on cells of normal liver tissue cell line THLE-3, thus linc-ITGB1 may be a safe therapeutic target for the treatment of HCC.

## Conclusion

linc-ITGB1 was up-regulated in HCC, and linc-ITGB1 overexpression may participate in the regulation of tumor growth and distant tumor metastasis. The role of linc-ITGB1 in HCC is likely achieved by up-regulating ROCK1. Our data suggest that linc-ITGB1 may serve a diagnostic marker and therapeutic target for HCC.

The article "Long non-coding RNA linc-ITGB1 promotes cell proliferation, migration, and invasion in human hepatoma carcinoma by up-regulating ROCK1" was retracted in 2023. Reasons: errors in the materials; concerns about the data.

## Abbreviations

CCK-8: Cell Counting Kit-8
DMEM: Dulbecco’s Modified Eagle Medium
GAPDH: Glyceraldehyde-3-phosphate dehydrogenase
ITGB1: Integrin beta-1
HCC: human hepatoma carcinoma
HRP: horseradish peroxidase
lncRNA: long non-coding RNA
LSD: least significant difference
OD: optical density
qRT-PCR: quantitative real time polymerase chain reaction
ROCK: Rho-associated, coiled-coil-containing protein kinase 1
TBST: tris-buffered saline tween
